# Helminth Communities of Owls (Strigiformes) Indicate Strong Biological and Ecological Differences from Birds of Prey (Accipitriformes and Falconiformes) in Southern Italy

**DOI:** 10.1371/journal.pone.0053375

**Published:** 2012-12-31

**Authors:** Mario Santoro, Simonetta Mattiucci, Giuseppe Nascetti, John M. Kinsella, Francesca Di Prisco, Sabatino Troisi, Nicola D’Alessio, Vincenzo Veneziano, Francisco J. Aznar

**Affiliations:** 1 Department of Public Health and Infectious Diseases, Section of Parasitology, Sapienza University of Rome, Rome, Italy; 2 Department of Ecological and Biological Sciences, Tuscia University, Viterbo, Italy; 3 Helm West Laboratory, Missoula, Montana, United States of America; 4 Istituto Zooprofilattico Sperimentale del Mezzogiorno, Section of Avellino, Monteforte Irpino, Avellino, Italy; 5 Istituto Gestione della Fauna Onlus, Naples, Italy; 6 Department of Pathology and Animal Health, University of Naples Federico II, Naples, Italy; 7 Instituto Cavanilles de Biodiversidad y Biología Evolutiva, y Departamento de Zoología, Universitat de València, Valencia, Spain; University of Western Ontario, Canada

## Abstract

We compared the helminth communities of 5 owl species from Calabria (Italy) and evaluated the effect of phylogenetic and ecological factors on community structure. Two host taxonomic scales were considered, i.e., owl species, and owls *vs*. birds of prey. The latter scale was dealt with by comparing the data here obtained with that of birds of prey from the same locality and with those published previously on owls and birds of prey from Galicia (Spain). A total of 19 helminth taxa were found in owls from Calabria. Statistical comparison showed only marginal differences between scops owls (*Otus scops*) and little owls (*Athene noctua*) and tawny owls (*Strix aluco*). It would indicate that all owl species are exposed to a common pool of ‘owl generalist’ helminth taxa, with quantitative differences being determined by differences in diet within a range of prey relatively narrow. In contrast, birds of prey from the same region exhibited strong differences because they feed on different and wider spectra of prey. In Calabria, owls can be separated as a whole from birds of prey with regard to the structure of their helminth communities while in Galicia helminths of owls represent a subset of those of birds of prey. This difference is related to the occurrence in Calabria, but not Galicia, of a pool of ‘owl specialist’ species. The wide geographical occurrence of these taxa suggest that local conditions may determine fundamental differences in the composition of local communities. Finally, in both Calabria and Galicia, helminth communities from owls were species-poor compared to those from sympatric birds of prey. However, birds of prey appear to share a greater pool of specific helmith taxa derived from cospeciation processes, and a greater potential exchange of parasites between them than with owls because of phylogenetic closeness.

## Introduction

In the last 30 years a number of papers on helminths of European owls (Strigiformes) have been published [1], [2], [3], [4], [5], [6], [7] including an exhaustive review of endoparasites found worldwide in raptors [8]. Most of those papers listed the helminth species identified and reported on basic statistical parameters of infection. When most than one owl species was studied from the same area, few attempts were made to investigate statistical differences between hosts and/or the factors influencing their helminth communities. Sanmartín et al. [7] concluded that in Galicia (northwest Spain) the helminth community of owls represented basically a “subset” of that observed in the birds of prey (Accipitriformes and Falconiformes) from the same region. This observation would agree with the observation that owls and birds of prey, although phylogenetically not closely related, have similar ecological niches and food habits, dividing the habitat not spatially but temporally [9]. Accordingly, their helminth faunas would be expected to be quite similar [10]. However, this prediction is at odds with the observed differences in composition of parasite faunas in geographical regions other than Galicia, i,e., Florida (USA) and Catalonia (northeast Spain), where a sizeable part of the faunas of each raptor group is not shared [6], [10], [11], [12], [13], [14]. These observations would therefore suggest that host specificity may play a contrasting role in structuring parasite communities in each raptor group depending on the geographical region.

Sanmartín et al. [7] also noted that helminth species richness of owl species was lower than that from birds of prey, and this result was considered unexpected given the similarity in hosts’ dietary spectrum. Ferrer et al. [6], [14] also indicated that, in Catalonia, owls exhibited lower diversity of helminths than birds of prey, and a similar conclusion can be derived from data by Kinsella et al. [10], [11], [12], [13] from Florida when values of helminth species richness are corrected for host sample size (MJ Kinsella, unpub. data). In attempting to account for these differences between raptor groups, Sanmartín et al. [7] suggested that a different explanation than feeding habits should be investigated. In this context, Kinsella et al. [10] pointed out body size as a potential determinant of helminth diversity among owl species; in fact, body size often correlates with key variables that affect transmission, i.e. host’s population density, rate of food intake or dietary breath ([15], [16] and references therein). The question is therefore whether body size could also help explaining the apparent differences in helminth richness between owls and birds of prey.

In southern Italy, Strigiformes include at least 7 species, displaying a wide variety of ecological and life-history patterns, including biological, environmental and dietary requirements [17]. In a recent published study from Calabria we found significant differences in both diversity and composition among helminths communities of 5 species of birds of prey [18]. Because several intrinsic and extrinsic factors including host age, sex, size, diet, habitat, behavior, migration, distribution and geographical range have all been recognized as variables influencing richness and diversity of parasite communities [18], [19], [20], [21], [22], [23], [24], [25], [26], [27], [28], we used a large sample of owl carcasses from southern Italy to evaluate the relative importance of the above mentioned variables on host biology, ecology and phylogeny on the structure of host-parasite associations at two taxonomical scales, i.e., between owl species, and between owls and birds of prey. The analysis benefits from the putative similarity in the regional pool of parasite species and the overall environmental characteristics from where owls and birds of prey were obtained.

Here we studied the helminth community of 5 owl species in Italy investigating the factors which may influence their community structure and comparing patterns of diversity and composition with those obtained among birds of prey from the same geographical area [18]. In addition, we evaluated overall differences in richness and the composition of helminth communities of owls and birds of prey, and compared the results with those previously obtained in Galicia [7]. The analyses were driven by the following research questions: (i) do the helminth communities of owl species from Calabria exhibit the same variability in composition and structure as that observed between birds of prey from the same region [18]? (ii) Are the helminth species from owls in Calabria “a subset” of the species found in birds of prey? (iii) Do owls have a lower diversity of helminth richness than birds of prey? (iv) What factors might account for the similarities and differences at each host’s taxonomical scale? And finally, do host body size play a role as an explaining factor?

## Materials and Methods

### Data Collection

A total of 122 owls that died between January 2004 and December 2011 at the Wildlife Rescue Centre in Rende, Cosenza (Calabria region), in southern Italy, were examined for helminth parasites. The birds belonging to 5 species of strigiforms including 30 little owls *Athene noctua*, 31 tawny owls *Strix aluco*, 41 barn owls *Tyto alba*, 10 long-eared owls *Asio otus*, and 10 scops owls *Otus scops* were all from the Calabria region. All owls included in the present study had a clinical course less than 7 days to minimize parasite losses; and no anthelmintic treatments were used in these birds [18], [27], [29].

All owl individuals were weighed prior to parasitological analysis. During necropsy examination, the trachea, lungs, air sacs, kidneys, spleen, liver, gallbladder, and the whole digestive tract of birds including oesophagus, stomach and intestines (duodenum, jejuno-ileum, ceca, and cloaca) were examined and helminths were collected, counted and identified following the techniques by Krone [30]. Worms were washed in saline solution and fixed in 70% ethanol; trematodes and cestodes were stained with Mayer’s acid carmine and mounted in Canada balsam, and nematodes and acanthocephalans were cleared in lactophenol on a glass slide for identification and then returned to the preservative. Voucher specimens are deposited in the U.S. National Parasite Collection, Beltsville, Maryland (Accession numbers: 105610 to 105625).

The whole pectoral muscles (depending by owl species approximately from 2 to 15 grams) and an aliquot of leg muscles (approximately from 2 to 5 grams) from each bird were examined for *Trichinella* spp. by artificial pepsin digestion [31].

### Comparison between Owl Species

Total abundance, species richness, Brillouin’s index of diversity, and the Berger-Parker dominance index were used as overall descriptors of infracommunities. Total abundance is the number of individuals of all helminth species, and species richness the number of helminth species, harbored by each individual owl. The 95% confidence interval (CI) for prevalence was calculated with Sterne’s exact method [32], and for mean values of intensity, total abundance, species richness, Brillouin’s index, and Berger-Parker index, with the bias-corrected and accelerated bootstrap method using 20,000 replications [33].

For each owl species, differences of total abundance, species richness, Brillouin’s index, and Berger-Parker index between genders were compared with Mann–Whitney U- tests, respectively. These parameters were also compared between owl species with Kruskal-Wallis tests using post hoc comparisons [34]. Inferential statistics on compositional differences between owl species were carried out with a nonparametric analysis of similarities (ANOSIM) [35]. The number of individuals of each helminth species from each infracommunity was square-root transformed, and the Bray-Curtis similarity coefficient was calculated between individual hosts that harbored at least 1 helminth species. The ANOSIM ranks the Bray-Curtis similarity matrix and tests whether the ranks of similarities between and within owl species are the same on average. This is evaluated with the statistic R [35]. The null hypothesis was constructed by calculating 20,000 R values with random permutation on host individuals regardless of species. The overall comparison was followed by pairwise comparisons between host species. When significant differences were found, the Similarity Percentage (SIMPER) procedure was used for assessing which helminth taxa were primarily responsible for the observed differences between groups [35].

### Compositional Differences of Helminth Faunas between Owls and Birds of Prey

Helminth data from the owl species analyzed in this study were compared with those obtained from 6 species of birds of prey examined by us in the same recovery centre between January 2000 and December 2010, i.e., 35 Eurasian buzzards *Buteo buteo*; 20 European sparrow hawks *Accipiter nisus*; 21 western honey buzzards *Pernis apivorus*; 17 marsh harriers *Circus aeruginosus*; 25 common kestrels *Falco tinnunculus*, and 17 peregrine falcons *Falco peregrinus* [18].

In Galicia, Sanmartín et al. [7] published infection data from 10 birds of prey species (110 Eurasian buzzards; 35 European sparrow hawks; 21 northern goshawks *Accipiter gentilis*; 12 common kestrels; 5 Montagu's harrier *Circus pygargus*; 3 western honey buzzards, 3 Eurasian hobbies *Falco subbuteo*; 2 peregrine falcons; 1 red kite *Milvus milvus* and 1 black kite *Milvus migrans*) and 4 owl species (49 barn owls, 26 tawny owls, 9 little owls and 8 long-eared owls) that were collected in four recovery centers from 1991 to 1996. This dataset provide a unique opportunity to replicate the above comparisons between owls and birds of prey in another geographical region.

To examine compositional differences between owls and birds of prey, prevalence values for each helminth species scaled to unity were used to obtain a matrix of similarities between raptor species using the Bray-Curtis coefficient. The resulting matrix was used to perform a group average hierarchical cluster of owl and birds of prey species [18]. To examine for statistical evidence of genuine clusters among species, 20,000 random permutations of prevalence values were employed in the matrix [35]. The finding of statistically significant clustering could assist in interpreting whether phylogenetic, and/or ecological, relatedness between raptor species could influence the similarity between their helminth faunas.

To interpret differences in overall composition of helminth faunas of owls compared to birds of prey we derived a measure of specificity for each helminth species found in the samples of owls from both Calabria and Galicia based on records on each species worldwide. For each helminth species we checked all references for synonymies and looked for taxonomic updates, assuming that original identifications were correct. Then, we established the following categories: a helminth species was considered ‘specialist’ if it had been reported in single host species; ‘owl specialist’ if it had been reported mainly, or only, in owls (Strigiformes); ‘birds of prey specialist’, if it had been reported mainly, or only, in birds of prey (Accipitriformes and Falconiformes); ‘raptor generalist’, if it had extensively been reported in both owls and birds of prey, and ‘bird generalists’, if it also occurred extensively in birds other than raptors. The use of host-parasite lists may suffer from well-known problems of representativity ([36], and references therein), namely, records may equate common and rare species, and suitable and unsuitable hosts (i.e., nonhosts). Therefore, estimations of the degree of specificity are conservative. For each helminth species, data were also gathered about its geographical distribution and the intermediate/paratenic hosts, which may assist in interpreting patterns of specifity and geographical differences in helminth faunas, respectively.

### Diversity differences of Helminth Communities between Owls and Birds of Prey

At the component community level (i.e., helminth communities for each host species considering the sample of hosts as a whole), we compared differences of species richness between owls and birds of prey from Calabria with an ANCOVA, considering the number of helminth taxa in each host species as the dependent variable, ‘raptor group’ as a fixed factor and ‘sample size’ (log_10_-transformed) as a covariate that correct for differences in sampling effort [22]. We firstly included the interaction term ‘raptor group×sample size’, but when it was not statistically significant, it was removed from the final model to increase the sensitivity of the analysis and to correctly interpret main effects [37]. The same ANCOVA analysis was carried out at infracommunity level, using data of mean species richness per host. Also, we investigated whether overall parasite recruitment differed between owls and birds of prey. Mean total abundance was discarded as an index of recruitment per host species because some small parasites (e.g., digeneans) were more numerous in birds of prey [18] and would strongly influence overall values. Instead, we calculated, for each host species, the median value of mean intensity of all parasites in the community since medians are very resistant to extreme values. This parameter was included as the dependent variable of an ANCOVA with the same predictors above.

We performed the same analyses described above with the data set from Galicia. For the comparison at the infracommunity analysis, Sanmartín et al. [7] only provided data for species with n≥8. Also, these authors did not provide values of mean species richness per host, but this value can easily be calculated for each host species as the sum of prevalences expressed on a per unit basis [38].

Effects of host body size upon community were explored as follows. Weight data from all raptor species included in the study were obtained from Snow et al. [39], and mean values for males and females throughout all seasons was averaged to obtain a single value per species. Then, for bird samples of both Calabria and Galicia, we examined whether residuals of component community richness, infracommunity richness, and the median value of mean intensity of all parasites in the community, corrected for host sample size, increased with host weight. One-tailed Spearman correlation tests were used. The package Primer v.6 [35] was used for the ANOSIM and cluster analyses, the free software Quantitative Parasitology v. 3 [40] to set 95% confidence intervals, and the statistical package SPSS v. 17 for the remaining analyses. Statistical significance was set at P<0.05.

## Results

### Comparison between Owl Species

A total of 19 helminth taxa (10 nematodes, 3 acanthocephalans,3 cestodes and 3 digeneans) and 758 helminth individuals were found in the total sample of owls (Table 1). All helminth taxa were found in the gastrointestinal tract except for a single specimen of *Excisa excisiformis* which was collected from the trachea of 1 long-eared owl. No *Trichinella* infection was found by artificial pepsin digestion of muscular tissues. Gravid individuals were found in all helminth taxa regardless of owl species. The total species richness in the sample ranged from 2 (in the long-eared owl) to 12 (in the tawny owl) (Table 1). No helminth species was shared between the 5 owl species, but *Centrorhynchus aluconis* and *Synhimantus affinis* were shared between 4 owl species. *Centrorhynchus aluconis* was also the most frequent species in little owls, tawny owls and barn owls, whereas *S. affinis* was the most prevalent species in scops owls (Table 1). Four helminth species were shared between 3 owl species and, as many as 12 helminth species were restricted to single owl species (Table 1). However, this restriction was not coupled with high specificity because, within this group, only *Paruterina candelabraria* and *Choanotaenia littoriae* is specific to a single owl species (Table 2), and prevalences were low or very low for all helminth species of this group (range: 3.2–20%, see Table 1).

**Table 1:** Infection parameters of helminths found in 5 species of owls from Calabria (southern Italy).

Helminth taxon		*Athene noctua*			*Strix aluco*			*Otus scops*			*Asio otus*			*Tyto alba*		
		(*n = *30)			(*n = *31)			(*n = *10)			(*n = *10)			(*n = *41)		
	P		I	P		I	P		I	P		I	P		I	
Acanthocephala																
*Centrorhynchus aluconis*	50.0 (32.4–67.6)		6.5 (3.5–12.7)	35.5 (20.7–53.3)		13.2 (5.6–25.7)	20 (3.7–55.4)		3.5 [2]–[5]	–		–	9.8 (3.4–22.9)		1.5 (1.0–1.8)	
*C. clitorideus*	6.7 (1.2–21.3)		8.5 [2]–[15]	–		–	–		–	–		–	–		–	
*C. globocaudatus*	–		–	3.2 (0.2–17.2)		1	–		–	–		–	–		–	
Nematoda																
*Capillaria falconis*	3.3 (0.2–17.7)		1	–		–	–		–	–		–	–		–	
*Heterakis gallinarum*	–		–	3.2 (0.2–17.2)		1	–		–	–		–	–		-	
*Dispharynx nasuta*	3.3 (0.2–17.7)		1	–		–	30.0 (8.7–61.9)		6.0 (4.0–7.3)	–		–	2.4 (0.1–13.0)		8	
*Hamatospiculum* sp.	–		–	3.2 (0.2–17.2)		5	–		–	–		–	–		–	
*Synhimantus affinis*	13.3 (4.7–29.8)		8.5 (3.0–10.8)	3.2 (0.2–17.2)		2	40.0 (15.0–70.9)		13.0 (4.0–29.5)	–		–	4.9 (0.8–16.7)		6.5 [3]–[10]	
*S. laticeps*	6.7 (1.2–21.3)		1.5 [1]–[2]	–		–	–		–	10.0 (0.5–44.6)		12	7.3 (2.0–19.3)		13.7 (1.0–26.0)	
*Skrjabinura spiralis*	–		–	–		–	20.0 (3.7–55.4)		1 [1]	–		–	–		–	
*Excisa excisiformis*	–		–	–		–	–		–	10.0 (0.5–44.6)		1	–		–	
*Porrocaecum spirale*	–		–	9.7 (2.7–25.5)		2.7 (2.0–3.3)	–		–	–		–	–		–	
*Subulura* sp.	–		–	3.2 (0.2–17.2)		1	10.0 (0.5–44.6)		1	–		–	–		–	
Digenea																
*Brachylaima fuscatum*	10 (2.8–26.3)		9.3 (3.0–13.7)	6.5 (1.2–20.7)		1.5 [1]–[2]	–		–	–		–	2.4 (0.1–13.0)		2	
*Neodiplostomum japonicum*	6.7 (1.2–21.3)		16 [14]–[18]	19.4 (8.8–36.9)		32.5 (14.5–68.8)	–		–	–		–	2.4 (0.1–13.0)		2	
*Skrjabinus* sp.	–		–	3.2 (0.2–17.2)		1	–		–	–		–	–		–	
Cestoda																
*Passerilepis stylosa*	–		–	3.2 (0.2–17.2)		8	–		–	–		–	–		–	
*Paruterina candelabraria*	–		–	9.7 (2.7–25.5)		5.7 (2.0–8.7)	–		–	–		–	–		–	
*Choanotaenia littoriae*	–		–	–		–	10.0 (0.5–44.6)		37	–		–	–		–	

P: prevalence (percentage of infected birds, %); I: mean intensity (mean number of worms per infected bird). *n* is the host sample size; numbers in parentheses are the 95% confidence intervals (C.I.) of each parameter. However, C.I. of mean intensity could not be calculated when the number of infected hosts was 1 or 2. In the latter case, the range of intensities is given in brackets.

**Table 2:** Classification of helminth taxa collected from owls in Calabria (C), southern Italy, and Galicia (G), northwest Spain, according to host specificity.

Helminth taxon	Hostrecords^1^	Geographical distribution	Specialist	Owls specialist	Birds of preys specialist	Raptor generalist	Bird generalist	No. hosts species infected	IH/PH
*Centrorhynchus aluconis*	A: Ag, Ar, Bb, Bl, Ca, Cc, Ha, Mmi	Europe, Asia				x		4 (C)	Orthopterans, terrestrial isopods/small mammals, reptiles
	F: Fn, Ft								
	S: Ao, Bbu, Os, Sa, Sur								
*C. clitorideus*	**S**: Ab, An, Os, Ta	Europe, Asia		x				1 (C)	Orthopterans, terrestrial isopods/small mammals, reptiles
*C. globocaudatus*	A: Ag, Apo, Bb, Bl, Br, Ca, Cc,Cp, Mm	Europe, Asia, Africa				x		1 (C) 3 (G)	Orthopterans, terrestrial isopods/small mammals, reptiles
	F: Fa, Fc, Fn, Fp, Ft, Fv								
	S: Af, Ao, An, Gp, Ns, Sa, Ta								
*Capillaria falconis*	A: Ag, An, Apo, At, Bb, Bj, Bl, Bli, Ha, Hl, Ph	Europe, Asia, North America				x		1 (C)	Earthworms
	F: Fs, Ft								
	S: Aa, Af, Ao, An, Bbu, Bv, Sa, So, Sv								
*C. tenuissima*	A: Ag, An, Bb, Bl, Cp, Ha, Mc, Mm, Mmi	Europe, Asia, South America				x		4 (G)	Earthworms
	F: Ft								
	S: Af, Afu, Ao, An, Bbu, Bv, Ns, Osu, Sa, Su, Sv, Ta								
*Excisa excisiformis*	S: Ao, Bv, Oa, Os, Sv	Europe, Asia, North America		x				1 (C)	?
*Hamatospiculum* sp.^2^						x?		1 (C)	?
*Heterakis gallinarum*	In at least 6 bird orders						x	1 (C)	Direct (facultative: earthworms and houseflies)
*Dispharynx nasuta*	In at least 10 bird orders						x	3 (C)	Terrestrial isopods
*Porrocaecum spirale*	A: Cp,	Europe, Asia, North America					x	1 (C)	Small mammals, reptiles
	F: Ft								
	S: Af, Afu, Ao, An, Bb, Bv, Ns, Sa, Su, Sur, Ta								
*P. angusticolle*	S: Ac, Ach, Ag, An, Apo, Ar, As, Bb, Bj, Bl, Bp, Ca, Cc, Cg, Ec, Ha, Hi, Mm, Mmi, Pa, Ph	Europe, Asia, North America			x			2 (G)	Earthworms/insectivors
	F: Fb, Fc, Fn, Fp, Fs Ft								
	S: Ao, Ta								
*Procyrnea leptoptera*	A: Ag, An, Bb, Bm, Bme, Bb, Gc, Hd, Mm, Mmi, Pa	Europe, Asia, South America			x			1 (G)	Orthopterans, coleopterans
	F: Fs, Fsp, Fn, Ft, Mc, Pp								
	S: Ta								
*Skrjabinura spiralis*	In at least 5 bird orders						x	1 (C)	?
*Subulura* sp.^3^							x?	2 (C)	?
*Synhimantus affinis*	S: Af, Ao, Bbu, Bv,Ta	Europe, North America		x				4 (C)	Terrestrial isopods, odonates, dermapterans/lizards?
*S. laticeps*	A: An, Ap, Bb, Bl, Ca, Cc, Cg, Cp, Mm, Mmi, Np, Pa	Europe, Asia, North America				x		3 (C) 3 (G)	Terrestrial isopods, odonates, dermapterans/lizards?
	F: Fc, Fco, Fn, Fp, Fs, Ft								
	S: Af, Ao, Bbu, Bv, Sa, Ta								
*Brachylaima fuscatum*	In at least 8 bird orders						x	3 (C)	Terrestrial snails
*Neodiplostomum japonicum*	S: Ao, Bbu	Italy, Japan		x				3 (C)	Freshwater snails, amphibians, reptiles (?)
*N. attenuatum*	A: Aco, Ag, As, Bb, Bj, Bli, Bp, Ca, Ef, Hl, Mm				x			4 (G)	Freshwater snails, amphibians, reptiles
	S: Sa, Su								
*Skrjabinus* sp.							x	1 (C)	Terrestrial mollusks, arthropods
*Strigea falconis*	A: Ac, Ach, Aco, Ag, Ah, Am, An, Ap, As, Apo, Ar, Bb, Bj, Bl, Bp, Cg, Ca, Cc, Cm, Cme, Cp, Ha, Mm, Mmi, Np, Ph, Pa, Te	Europe, Asia, America, Africa				x		1 (G)	Aquatic snails, amphibians, reptiles, birds, small mammals
	F: Fb, Fc, Fco, Fn, Fp, Fs, Fsp, Ft, Fv								
	S: Af,Ao, Bbu, Bv, Sa, Su, Sv, Ta								
*Choanotaenia littoriae*	S: An	Italy	x					1 (C)	Insects
*Paruterina candelabraria*	S: Ao, Bv, Ns, Os, Sa, Su	Europe, North America		x				1 C, 1 G	Insects, rodents
*Passerilepis stylosa*	Typical from Passeriformes						x	1 C	Insects

Classification is based on global records of host species for each helminth taxon ([63], [64], [65], [66], [67], [68] and references detailed in the text); data about the geographical distribution of helminth taxa typical from raptors is also listed. Specificity categories are defined in the text. For each helminth taxon, information is also provided about its known or putative intermediate/paratenic hosts (IH/PH) and the number of owl species it infects in Calabria and/or Galicia.

1 Host species abbreviations:

Accipitriformes (A): Ac: *Aquila clanga*; Ach, *Aquila chrysaetos*; Aco, *Accipiter cooperi*; Ag, *Accipiter gentilis*; Agu, *Accipiter gularis*; Ah, *Aquila heliaca*; Am, *Aegypius monachus*; An, *Accipiter nisus*; Ap, *Aquila pennata*; Apo, *Aquila pomarina*; Ar, *Aquila rapax*; As, *Accipiter striatus*; At, *Accipiter trivirgatus*; Bb, *Buteo buteo*; Bj, *Buteo jamaicensis*; Bl, *Buteo lagopus*; Bli, *Buteo lineatus*; Bm, *Buteo magnirostris*; Bme, *Buteogallus meridionalis*; Bp, *Buteo platypterus*; Br, *Buteo rufinus*; Ca, *Circus aeruginosus*; Cc, *Circus cyaneus*; Cg, *Circaetus gallicus*; Cm, *Circus macrourus*; Cme: *Circus melanoleucos*; Cp, *Circus pygargus*; Ec, *Elanius caeruleus*; Ef, *Elanoides furficatus*; Gc, *Geranospiza caerulescens*; Ha, *Haliaeetus albicilla*; Hd, *Harpagus diodon*; Hi, *Haliastur indus*; Hl, *Haliaeetus leucophalus*; Mc, *Milvago chimango*; Mm, *Milvus milvus*; Mmi, *Milvus migrans*; Np: *Neophron percnopterus*; Pa, *Pernis apivorus*; Ph, *Pandion haliaetus*; Te, *Theratopius ecaudatus.*

Falconiformes (F): Fa: *Falco ardosiaceus*; Fb, *Falco biarmicus*; Fc, *Falco cherrug*; Fco, *Falco columbarius*; Fn, *Falco naumanni*; Fp, *F. peregrinus*; Fs, *Falco subbuteo*; Fsp, *Falco sparverius*; Fr: *Falco rufigularis*; Ft, *F. tinnunculus*; Fv, *Falco vespertinus*; Mc, *Milvago chimachima*; Pp, *Polyborus plancus.*

Strigiformes (S): Aa, *Aegolius acadicus*; Ab, *Athene brama*; Af, *Asio flammeus*; Afu, *Aegolius funereus*; An, *Athene noctua*; Ao, *Asio otus*; Bbu, *Bubo bubo*; Bv: *Bubo virginianus*; Gp, *Glaucidium passerinum*; Ns, *Nyctea scandiaca*; Oa: *Otus asio*; Os, *Otus scops*; Osu, *Otus sunia*; Sa, *Strix aluco*; So, *Strix occidentalis*; Su, *Surnia ulula*; Sur, *Strix uralensis*; Sv, *Strix varia*; Ta, *Tyto alba.*

2 Most species are typical from birds of prey.

3 Two species are specific to owls.

The proportion of individual hosts that were infected in the sample differed significantly among host species (Fisher test, p<0.003), ranging from 2 out of 10 (10%) in long-eared owls to 7 out of 10 (70%) in scops owls (Table 3). Infracommunity parameters for each host species are shown in Table 3. There were no significant differences in mean species richness (Kruskal-Wallis test, χ^2^ = 8.64, 4 d.f., p = 0.071), mean total abundance (χ^2^ = 7.11, 4 d.f., p = 0.130) and Brillouin’s diversity index (χ^2^ = 2.71, 4 d.f., p = 0.607) of helminths between owl species. The Berger-Parker index did not differ also between owl species (χ^2^ = 6.68, 4 d.f., p = 0.154) and the most abundant helminth species in infracommunities accounted for a very high proportion of total helminth abundance (mean Berger-Parker index >0.80 in all host species, Table 3). *Centrorhynchus aluconis* was numerically dominant in little owls, tawny owls and barn owls (in the latter shared with *S. laticeps*), whereas *S. affinis* was dominant in scops owls and *Synhimantus laticeps* in long-eared owls (shared with *E. excisiformis*) (Table 3). Mean similarity values of helminth infracommunities between owl species are shown in Table 4. Similarities ranged from 33.6% to 51.5%. Note that only 2 long-eared owls were infected (Table 3) and, therefore, comparisons with the other species are uncertain. Overall, helminth infracommunities of scops owls had the lowest similarity with those from the remaining species (Table 4). Statistical comparison of compositional differences between owl species (excluding the long-eared owl) revealed modest, but significant differences of composition among owl species (ANOSIM, R = 0.173, p = 0.0005). Two pairwise comparisons were found to be significant, namely, those involving scops owls and little owls (R = 0.402, p = 0.004), and scops owls and tawny owls (R = 0.338, p = 0.002); the comparison between scops owls and barn owls was close to significance (R = 0.162, p = 0.059). In the two significant comparisons, *C. aluconis* and *S. affinis* ranked as the first and second species providing dissimilarity between owl species according to The SIMPER procedure. Together, these 2 species accounted for 48.7% (scops owls *vs.* little owls) and 38.9% (scops owls *vs.* tawny owls) of mean dissimilarity. We found no statistically significant effects of host weight (Spearman correlation test, minimum nominal p = 0.145) or sex (Mann-Withney test, minimum nominal p = 0.183) on any 4 infracommunity parameters of Table 3 for any owl species. In the case of long-eared owls the tests involving Brillouin’s diversity index and Berge-Parker index could not be performed because only 2 hosts were infected (Table 3).

**Table 3:** Mean values (95% C.I.) of 4 parameters of gastrointestinal helminth communities in 5 owl species in Calabria (southern Italy).

Host species	Mean weight (S.D.) (g)	Species richness	Total abundance	Brillouin index	Berger-Parker index	Dominant species
*Athene noctua*	103.8 (23.3)	1.00 (0.63–1.33)	7.1 (4.1–12.2)	0.25 (0.13–0.39)	0.83 (0.73–0.91)	*C. aluconis* [66.7]
(*n* = 30, 18 infected)						
*Strix aluco*	203.3 (28.7)	1.03 (0.65–1.45)	12.5 (6.6–22.9)	0.21 (0.10–0.37)	0.89 (0.80–0.95)	*C. aluconis* [44.4]
(*n* = 31, 18 infected)						
*Otus scops*	43.7 (7.9)	1.30 (0.60–1.80)	11.7 (3.9–25.0)	0.28 (0.10–0.46)	0.83 (0.68–0.94)	*S. affinis* [57.1]
(*n* = 10, 7 infected)						
*Asio otus*	218.5 (50.8)	0.20 (0.00–0.40)	7.1 (4.2–11.9)	0	1.0	*S. laticeps* [50.0]
(*n* = 10, 2 infected)						*E. excisiformis* [50.0]
*Tyto alba*	203.3 (28.7)	0.29 (0.15–0.46)	1.8 (0.4–6.6)	0.07 (0.00–0.19)	0.97 (0.87–0.98)	*C. aluconis* [30.0]
(*n* = 41, 10 infected)						*S. laticeps* [30.0]

The parasite taxa that are more frequently dominant in the infracommunities for each host species are also reported. Numbers in brackets are the percentage of hosts in which each parasite taxon is dominant.

**Table 4:** Matrix of mean values (with standard devistion in parentheses) of Bray-Curtis index of similarity (expresed as percentage) of helminth infracommunity composition between 5 owl species from the Calabria region, southern Italy.

	*Athene noctua*	*Strix aluco*	*Otus scops*	*Asio otus*
***Strix aluco***	49.1			
	(19.6)			
***Otus scops***	41.3	34.3		
	(16.5)	(12.8)		
***Asio otus***	37.0	34.6	33.6	
	(7.8)	(8.8)	(7.7)	
***Tyto alba***	51.5	44.0	42.6	47.9
	(21.8)	(17.3)	(17.3)	(15.5)

### Compositional Comparison of Helminth Communities between Owls and Birds of Prey

The group-average hierarchical cluster of raptor species based on prevalence of their helminth fauna is shown in Figure 1. In Calabria, a major significant subdivision (p = 0.0005) separated owls and birds of prey (Fig. 1A). However, in Galicia the cluster did not have any significant nodes, and species were not arranged according to the subdivision between owls and birds of prey.

**Figure 1:** Group-average hierarchical cluster analysis of helminth fauna from samples of birds of prey and owls in two geographical regions based on a bray-Curtis resemblance matrix using prevalence data scaled to unity. The number on the node indicates the probability that the node is random (see text for details). A. Calabria, Italy. B. Galicia, Spain.

Data about specificity of each helminth species are shown in Table 2. In Calabria, specificity could be established in 18 out of 19 helminth taxa, and they were distributed as follows: 1 species was classified as ‘specialist’; 6 as ‘owl specialists’, 5 as ‘raptor generalists’ and 6 as ‘bird generalists’. Species typical from owls (the two former categories) summed up 410 helminth individuals, or 54.1% of all helminth individuals found in the total sample of owls (see Table 1). In Galicia, 8 helminth species were reported, of which 1 species can be classified as ‘owl specialist’, 3 as ‘birds of prey specialists’, and 4 as ‘raptor generalists’. The single species typical from owls, *P. candelabria*, was found only in a single species (Table 2).

### Diversity differences of Helminth Communities between Owls and Birds of Prey

At the component community level, the ANCOVA for species richness indicated that the interaction between host sample size and raptor group was significant neither in Calabria nor in Galicia and, therefore, interactions were removed from the models. Host sample size had an overall significant positive effect on species richness (Calabria: F_(1,8)_ = 6.124, p = 0.038, Galicia: F_(1,11)_ = 26.532, p<0.001); differences between raptor groups were also significant in both regions (Calabria: F_(1,8)_ = 8.568, p = 0.019, Galicia: F_(1,11)_ = 8.602, p = 0.014), with birds of prey having higher values of species richness in their helminth communities (Fig. 2 A, B). At infracommunity level, the ANCOVA for mean species richness also revealed that the interaction between host sample size and raptor group was not significant in either region. Also, there were no significant effects of host sample size (Calabria: F_(1,8)_ = 0.001, p = 0.995, Galicia: F_(1,5)_ = 2.694, p = 0.162), although sample size in Galicia was very low (Fig. 2 C, D). Concerning raptor group, helminth infracommunities from birds of prey in Calabria had higher values that those from owls (Fig. 2C) and the difference was significant (F_(1,8)_ = 5.518, p = 0.045). In Galicia, this pattern was less marked (Fig. 2D) and the difference was not significant (F_(1,5)_ = 1.771, p = 0.241).

**Figure 2:** Comparison of community parameters between species of birds of prey (solid dots) and owls (empty dots) in two geographical regions, Calabria, Italy (on the left) and Galicia, Spain (on the right). A, B: Total species richness at the component community level. Regressions lines for birds of prey (solid lines) and owls (broken lines) are also displayed. C, D. Mean species richness at infracommunity level. Bars represent the 95% confidence interval. C, D. Median value of mean intensity per host species. The regressions line for birds of prey in Calabria is shown. Bars represent the interquartilic interval. Species abbreviations: *Ag*: *Accipiter gentilis*; *An*: *Athene noctua*; *Ani*: *Accipiter nisus*; *Ao*: *Asio otus*; *Bb*: *Buteo buteo*; *Ca*: *Circus aeruginosus*: *Cp*: *Circus pygargus*; *Fp*: *Falco peregrinus*; *Fs*: *Falco subbuteo*; *Ft*: *Falco tinnunculus*; *Mm*: *Milvus milvus*; *Mmi*: *Milvus migrans*; *Os*: *Otus scops*; *Pa*: *Pernis apivorus*; *Sa*: *Strix aluco*; *Ta*: *Tyto alba*.

The ANCOVA for the median values of mean intensity (MMI) also offered contrasting pattern between geographical regions. In Calabria, the interaction between host sample size and raptor group was significant (F_(1,7)_ = 11.861, p = 0.011). Apparently, host sample size influenced MMI only in birds of prey (Fig. 2E). Ignoring the effects of host sample size, the comparison of MMI between raptor groups was significant (F_(1,8)_ = 5.445, p = 0.048), and birds of prey tended to exhibit higher values of MMI. In Galicia, none of the predictors was significant (results not shown), and MMI was similar between owls and birds of prey (Fig. 2F). Host weight did not significantly correlate with host sample-size-corrected residuals of component community richness, mean infracommunity richness, and the median value of mean intensity of all parasites in the community either in Calabria or Galicia (Spearman correlation, all one-tailed p>>0.05).

## Discussion

### Comparison Among Owls Species

Because most of the helminths in birds are acquired through the ingestion of their prey, the overall environment with its included habitats influencing the survival and potential transmission of a parasite species have been considered as the most important extrinsic determinants of pattern in helminth communities of avian hosts [19], [23], [24], [28], [41]. Host vagility, a broad host diet, and selective feeding by a host on prey that serve as intermediate hosts for a wide variety of helminths represent the main intrinsic determinants influencing their helminth communities [19], [23], [24], [41].

Ecological determinants are important when considering the similarities and differences of helminth communities between owls in Calabria. Three types of helminth species can be recognized, namely, species typical from owls (including an apparently very specific species, *C. littoriae*), species shared also with birds of prey, and generalist parasites common to other birds. It is not possible to determine whether all owl species are equally suitable hosts for each of these parasites, but patterns of specificity, and the absence of significant subdivisions of owls in the cluster analysis, strongly suggest that there are not fundamental barriers for exchange of helminth taxa among owl species. Therefore, factors driving the contact between owls and parasites [16], especially diet [15] are predicted to mainly account for the similarities and differences in their helminth faunas.

The owl species here studied are crepuscular and nocturnal feeders. According to Snow et al. [39], in the western Palaearctic scops owls feed mostly on insects and other invertebrates, whereas the remaining species rely more on small mammals and other vertebrates. However, each owl species can adjust their diet according to local availability, including a variable portion of birds, reptiles, amphibians and invertebrates [39], [42], [43]. Unfortunately no studies on feeding ecology of owls were available from Calabria, but results from studies in other regions of Italy largely conform to the general pattern described above, with scops owls feeding mainly on insects (orthopterans and moths) [44], barn owls, tawny owls and long-eared owls feeding more on small mammals [45], [46], [47], and little owls having a mixed diet of insects and small vertebrates [48].

Statistical comparison of helminth communities in owls from Calabria showed only marginal differences between scops owls and little owls and tawny owls. These differences are largely accounted for variability of infection levels of 2 helminth species which account for over 80% of total helminth abundance, i.e., *C. aluconis* (higher in little owls and tawny owls) and *S. affinis* (higher in scops owls). *Centrorhynchus aluconis* is known to use a wide range of micro-mammals and reptiles as paratenic hosts [49], [50], [51] in which the parasite accumulates. The life cycle of *S. affinis* is not known, but data from allied species indicates that insects and terrestrial isopods act as intermediate hosts [52] and lizards could act as paratenic hosts [53]. We therefore interpret that the largely insectivorous diet of scops owls would led them to recruit more individuals of *S. affinis*, and less of *C. aluconis*, compared to the other owl species.

The otherwise strong similarities in community structure of helminth communities of owls from Calabria are in contrast to the strong differences observed in birds of prey from the same region. Santoro et al. [18] interpreted that these differences resulted from diverse feeding habits among hosts (e.g., insectivory in western honey buzzards, ornithophagy in peregrine falcons, or a more catholic diet in Eurasian buzzards). Conversely, we submit that the small differences found in owls would indicate that all the studied species feed on a narrower range of prey, consuming different proportions of invertebrates, micro-mammals, and small vertebrates depending on both species and local availability. For example, in Greece, the barn owl preyed mainly on mammals, while birds and amphibians were only of local importance, and, accordingly, diet showed low diversity; the long-eared owl preyed mainly on mammals, but also took other prey (particularly birds and reptiles)**,** having a more diverse diet. In contrast, the diet of the little owl was more variable, in two of the study areas the main prey were mammals but other prey involved resulted in relatively high diversity. In the other three areas the species took mainly insects, thus showing a more restricted diet based on small-sized prey [43]. In a study from Chile, Spain and California was observed that in Spain barn owl feed on significant amount of insects, reptiles and amphibians respect to those from Chile and California, and also the mean size of small mammals in its diet was considerably smaller than that from other two areas [42]. This was attributed to the reduced abundance of larger-sized small mammals in Spain, which presumably forces the barn owl to prey more heavily on the smallest mammals available and also on low-reward non-mammalian prey [42]. This suggests that owls may adapt their trophic requirements to the reduced prey occurring in a particular geographical area.

### Compositional Differences of Helminth Faunas between Owls and Birds of Prey

Cluster analysis indicated that, in Calabria, owls can be separated as a whole from birds of prey with regard to the structure of their helminth communities; no further subdivisions among owl species were significant. This pattern results largely from the occurrence of ‘owl specialist’ species, which account for over 50% of total helminth abundance. It is also important to note that owls and birds of prey share just 4 of the 50 helminth taxa found in total (19 in owls and 31 in birds of prey) showing different infection levels; shared parasites included *C. globocaudatus*, *C. falconis*, *S. laticeps*, and *B. fuscatum* (see [18], [26]). The first 3 parasite species are very common in birds of prey from southern Italy, while in owls had lower prevalence and intensity; and only immature *B. fuscatum* were found in birds of prey and mature specimens in owls, respectively [18], [26].

Interestingly, ‘owl specialists’ are species shared only among owls, not just in Calabria, but apparently throughout their entire geographical distribution. For instance, the cestode *P. candelabraria* has extensively been reported only in owl species from Europe and North America (Table 2). This raises the question of what factors could produce these patterns of specificity. The encounter/compatibility paradigm [54], [55] states that specificity is determined by two sequential filters. The encounter filter prevents infections of potential hosts that cannot contact the parasite, whereas the compatibility filter excludes contacted hosts in which the parasite is unable to find the appropriate resources and/or escape or deter the host’s defences. The compatibility filter is directly associated to the history of co-adaptation between parasites and their hosts, and predicts that hosts that are phylogenetically related will tend to share parasites, among other factors, because they have a similar physiology [16].

Because of the lack of information, it is difficult to assess the role of the encounter and compatibility filters in shaping specificity of the ‘owl specialist’ helminths that were found in Calabria. Does, for instance, *P. candelabraria* use intermediate and paratenic hosts that are consumed only by owls and/or is it specialized for the microhabitat conditions provided by owls as hosts? We noted above that no dietary data exists for owls in Calabria but, in general, owls foraging at dusk and during the night are predicted to encounter only certain prey compared to birds of prey which are diurnal predators feeding generally on a wider spectrum of prey. There is only a subset of prey whose active times overlap with that of the both raptor groups, which are the ones more likely to be caught by both of them [56], [57]. Therefore, owls and birds of prey might share a limited number of prey species, constraining exchange of parasites. However, it is likely that some ‘owl-specialist’ species that contact non-owl hosts are also unable to establish and reproduce in them. For example, in North America, *P. candelabraria* have been reported in shrews, deer mice, voles and squirrels [58], which are regularly consumed by birds of prey [59] but none of them has been reported as a host for *P. candelabraria*, suggesting that the parasite cannot established in them.

Four out of the 5 owls species (barn, long-eared, tawny and little owls) included in the present study were also examined for helminths in Galicia [7]. Interestingly, ‘owl specialists’ were missing in this sample except for *P. candelabraria*, and owls essentially harboured a subset of the helminths found in birds of prey [7] (Table 2). This striking difference in composition can hardly be related to biogeographical factors because ‘owl specialist’ species have generally very wide geographical distributions (Table 2). Alternatively, compositional variability might be related to differences in the local pool of parasites [16], [24]. In support of hypothesis, of 27 total helminths found in owls from Calabria (19) and Galicia (8) just 3 were common in both localities (Table 2). In fact, local variability seems to be a common theme in other geographical areas. In Netherlands, for instance, Borgsteede et al. [5] analyzed 84 owls of 5 species (including barn, long-eared, tawny and little owls) and identified 12 helminth species excluding cestodes, of which only *Porrocaecum spirale* can be considered as an ‘owl specialist’ (Table 2). The role of local conditions, especially the availability of intermediate and paratenic hosts cannot be overestimated in accounting for these local differences [16].

Of the helminths species found here, the nematodes including *Dispharynx* spp., *Excisa* spp., *Synhimantus* spp., *Skrjabinura* spp., and *Subulura* spp. use a wide range of insects as intermediate hosts, and *Capillaria falconis* and *Heterakis gallinarum* use earthworms; *Porrocaecum* spp. use insectivorous mammals [52]; cestodes within *Choanotaenia* spp. use coleopterans and dipterans, *Passerilepis* spp. use insects, and *P. candelabraria* uses micro-mammals [60]; among digeneans *Neodiplostomum* spp. use amphibians, *B. fuscatum* uses terrestrial snails [61] and *Skrjabinus* spp. use terrestrial mollusks and arthropods [62]; acanthocephalans within *Centrorhynchus* spp. use orthopteran insects as intermediate hosts and mammals, reptiles and anurans as paratenic hosts [49], [50], [51] (Table 2).

### Diversity Differences of Helminth Communities between Owls and Birds of Prey

The statistical comparison of diversity of helminth communities between owls and birds of prey assume that observations are independent. This is not the case because species within each bird group are related through phylogenetic relationships [15]. However, given the small sample of raptor species included in the study, our exploratory comparison was considered as a useful starting for future analyses that will include more raptor species and will explicitly control for phylogenetic effects ([15], and references therein). Currently, results indicate that the helminth fauna of owls from both Calabria and Galicia was less diverse than that from birds of prey in the same regions, thus statistically confirming conclusions previously obtained by Sanmartín et al. [7] for Galicia. The pattern could indeed be more general. In Catalonia, Ferrer et al. [6], [14] also observed that compared to birds of prey, owls had lower numbers of genera of helminths (14 vs 22), and generally lower prevalence rates among shared genera. Data from Kinsella et al. [10], [11], [12], [13] in Florida would also point to a similar conclusion when the effects of sampling effort are accounted for (MJ Kinsella, unpub. data). Overall, evidence would suggest that there are significant differences in the diversity of helmith faunas between owls and birds of prey regardless of the actual pool of species that can potentially infect host species in each region (see above). We therefore interpret that there might be a common factor producing this pattern.

A number of host-related factors have been put forward to account for differences in species richness of parasites among vertebrates, of which factors related to host body size often play a prominent role [15], [16], [23], [36]. Although our analyses should be interpreted with care because of small host sample sizes, host body size did not significantly correlate with species richness, neither at infracommunity nor at component community levels. Also, median intensity of helminths did not increase in large-bodied species, suggesting that the rate of parasite recruitment was not related to the amount of food consumed. Also, there was not an evident relationship between helminth infracommunity parameters and body size in owls (Table 3).

We suspect that other factors probably blur the expected influence of host body size upon helminth communities. One potential candidate is trophic niche breath [16]. Kinsella et al. [10] speculated that species richness in the helminth fauna of owls from Florida was primarily related to the variety of prey items consumed, with specialized feeders like barn owls and screech owls (*Otus asio*) harbouring fewer species than euryphagic species like barred owls (*Strix varia*). However, at a larger taxonomic scale, Sanmartín et al. [7] argued against a direct influence of diet because both owls and diurnal raptors share the same basic pool of prey in Galicia.

A factor missing in latter explanation is the influence of parasite specificity, which is much more apparent in birds from Calabria. In the previous section we pointed out that, regardless of contacts between parasites and hosts, the compatibility filter prevents some parasites from being established in certain hosts, but the filter should be more relaxed insofar as hosts species are phylogenetically closer. Accipitriformes plus Falconiformes represent a more speciose group than Strigiformes (ca. 58 vs. 19 spp., respectively, in the western Palaearctic, see Snow et al. [39]). It is therefore possible that birds of prey, as a group, harbor more specific helminth taxa than owls [8]. Also, the diversity of birds of prey generally outnumbers that of owls in any locality in Europe [39]. Following both arguments, we could expect, in any locality, that birds of prey share a greater pool of specific helmith taxa derived from cospeciation processes, and a greater exchange of parasites between them than with owls. The observation that both in Calabria and Galicia there are a number of helminth species shared between diurnal raptors with diverse trophic habits, but that do not occur in sympatric owls would lend support to this hypothesis. We urge researchers to develop specific analysis to test this hypothesis when more quantitative data about helminth communities from raptors are gathered in the future.
